The article "Melatonin attenuates acute kidney ischemia/reperfusion injury in diabetic rats by activation of the SIRT1/Nrf2/HO-1 signaling pathway" was published in 2019. Journal: Biosci Rep.

# Melatonin attenuates acute kidney ischemia/reperfusion injury in diabetic rats by activation of the SIRT1/Nrf2/HO-1 signaling pathway

**DOI:** 10.1042/BSR20181614

**Published:** 2019-01-15

**Authors:** Si Shi, Shaoqing Lei, Chaoliang Tang, Kai Wang, Zhongyuan Xia

**Affiliations:** 1 Department of Anesthesiology, Renmin Hospital of Wuhan University, Wuhan, Hubei, China; 2 Department of Anesthesiology, The First Affiliated Hospital of USTC, Division of Life Sciences and Medicine, University of Science and Technology of China, Hefei, Anhui, China

**Keywords:** diabetes, ischemia reperfusion injury, melatonin, silent information regulator 2 associated protein 1

## Abstract

**Background and aims:** Diabetic kidney is more sensitive to ischemia/reperfusion (I/R) injury, which is associated with increased oxidative stress and impaired nuclear factor erythroid 2-related factor 2 (Nrf2)/heme oxygenase-1 (HO-1) signaling. Melatonin, a hormone that is secreted with the rhythm of the light/dark cycle, has antioxidative effects in reducing acute kidney injury (AKI). However, the molecular mechanism of melatonin protection against kidney I/R injury in the state of diabetes is still unknown. In the present study, we hypothesized that melatonin attenuates renal I/R injury in diabetes by activating silent information regulator 2 associated protein 1 (SIRT1) expression and Nrf2/HO-1 signaling. **Methods:** Control or streptozotocin (STZ)-induced Type 1 diabetic rats were treated with or without melatonin for 4 weeks. Renal I/R injury was achieved by clamping both left and right renal pedicles for 30 min followed by reperfusion for 48 h. **Results:** Diabetic rats that were treated with melatonin undergoing I/R injury prevented renal injury from I/R, in aspects of the histopathological score, cell apoptosis, and oxidative stress in kidney, accompanied with decreased expressions of SIRT1, Nrf2, and HO-1 as compared with those in control rats. All these alterations were attenuated or prevented by melatonin treatment; but these beneficial effects of melatonin were abolished by selective inhibition of SIRT1 with EX527. **Conclusion:** These findings suggest melatonin could attenuate renal I/R injury in diabetes, possibly through improving SIRT1/Nrf2/HO-1 signaling.

## Introduction

Acute kidney injury (AKI) is a global public health problem that affects millions of people, and it has become increasingly prevalent in recent years [1]. Several risk factors such as age, race, genetic factors, hypertension, and diabetes are associated with AKI [1]. Diabetes is associated with a variety of metabolic disorders, such as hypoxia, overproduction of reactive oxygen species (ROS), mitochondrial dysfunction, and inflammation [2]. Moreover, diabetes is the major cause of chronic kidney disease in most developed countries [3]. Diabetic nephropathy (DN) is one of the serious organ complications of diabetes, and DN is the leading cause of end-stage renal disease (ESKD) in the world [2,4]. In diabetic kidney tissue, hyperglycemia can promote the production of ROS and increase the level of oxidative stress [5]. Animal model studies in rats confirmed that diabetic rats had increased vulnerability to renal ischemia/reperfusion (I/R) compared with normal rats [6,7]. However, the underlying mechanisms by which hyperglycemia adversely affects renal I/R in diabetes has remained elusive.

Melatonin is mainly produced by the pineal gland and it acts as a natural antioxidant and free radical scavenger [8–10]. Melatonin not only acts on ROS, reactive nitrogen species, and free radicals but also up-regulates antioxidant enzymes and down-regulates pro-oxidant enzymes [11–13]. Endogenous and exogenous melatonin can reduce diabetes-related metabolic disorders by regulating insulin secretion and scavenging ROS [14]. Chronic melatonin treatment reduces renal damage by restricting lipid oxidation and NO production in STZ-induced diabetic rats exposed to renal I/R [15]. In rat kidney transplantation model, melatonin protects kidney from I/R injury by down-regulating the expression of NF-kBp65, iNOS, and caspase-3 [16], while in the rat model of renal warm I/R, the melatonin signaling phosphorylated Akt, inhibited GSK-3β and VDAC [17]. Melatonin showed neuroprotective effects by activating nuclear factor erythroid 2-related factor 2 (Nrf2)/ARE pathway and increasing levels of antioxidant enzymes heme oxygenase-1 (HO-1) and NQO1 expression [18]. Although melatonin has both pro- and anti-inflammatory activities [19,20], the known protective effects of melatonin in I/R injury is primarily via its antioxidative stress rather than the pro-inflammatory cytokines [21,22].

Silent Information Regulator 2 Associated Protein 1 (SIRT1) is a deacetylase regulating the processes of aging, cancer, glucose metabolism, and energy homeostasis [23–25]. It is well described that SIRT1 reduces oxidative stress, inflammation stimuli, cell senescence, and apoptosis [26–32]. In addition, a study suggested that SIRT1 protects kidneys from renal damage in a melatonin-dependent manner in rats with severe burn-induced AKI rat model [33].

Nrf2 is a major transcriptional regulator of antioxidant proteins [34]. After cell injury, Nrf2 translocates to the nucleus and promotes the expression of HO-1 [35]. Several studies confirmed that SIRT1 could promote the activation of Nrf2, including increasing its nuclear accumulation, DNA binding activity, and transcriptional activity, and up-regulating the expression of HO-1 [36–38]. However, whether SIRT1 can attenuate renal I/R injury by activating the Nrf2/HO-1 signaling pathway in diabetes has not been reported. In the present study, we determined that melatonin activates the Nrf2/HO-1 signaling pathway by up-regulating the expression of SIRT1, thereby reducing diabetic renal I/R injury.

## Materials and methods

### Animals and reagents

Male adult Sprague–Dawley rats (250 ± 10 g, 6–8 weeks of age) were purchased from Beijing HFK Bioscience Co., Ltd. (Beijing, China). All rats were housed at 22–24°C, a 12-h light/dark cycle with free access to standard rat chow and water. The experimental protocols were in accordance with the principles of Animal Care of Wuhan University (Wuhan, China), and approved by the Ethics Committee of Renmin Hospital of Wuhan University. Streptozotocin (STZ) and melatonin were purchased from Sigma–Aldrich (St. Louis, MO, U.S.A.). EX527 was purchased from Selleck Chemicals (TX, U.S.A.). Primary antibodies against SIRT1 and HO-1 were purchased from Abcam, Inc. (Cambridge, U.K.). Primary antibodies against Nrf2 were purchased from Santa Cruz Biotechnology, Inc. (Dallas, TX, U.S.A.). Primary antibodies against GAPDH and Lamin B were purchased from Cell Signaling Technology, Inc. (MA, U.S.A.). Second antibodies were purchased from LI-COR Biosciences (IRDye 800CW; LI-COR Corporate, Lincoln, NE, U.S.A.).

### Induction of diabetes

Type 1 diabetes was induced by a single intraperitoneal injection of STZ solution dissolved in 0.1 M citrate buffer (pH 4.5) at a dose of 60 mg/kg body weight, as previously described [39]. Normal rats were given a single intraperitoneal of the same equal volume citrate buffer. Three days after STZ injection, tail vein blood glucose levels were measured with a One Touch Ultra Glucose meter (Johnson & Johnson, New Brunswick, NJ, U.S.A.). Only those rats with fasting blood glucose level ≥16.7 mM were considered as diabetic [39].

### Renal I/R injury model

Animals were intraperitoneally anesthetized by pentobarbital sodium (60 mg/kg body weight) and then placed on a homeothermic pad to maintain a core body temperature of 37°C. Kidneys were exposed by abdominal midline incisions, and both left and right renal pedicles were clamped for 30 min to induce ischemia. After ischemia, the clamps were released for 48 h reperfusion. The same procedure was performed in the nondiabetic control animals without the bilateral clamping process. The abdominal wall wounds were closed and rats intraperitoneally received 1 ml warm saline. All rats were killed by cervical dislocation after 48 h of reperfusion. Plasma and kidneys samples were collected and stored at −80° C for further analysis.

### Experimental protocol

At 4 weeks of diabetes, both diabetic and nondiabetic control rats were randomly allocated into six groups of 6–8 rats each: (i) nondiabetic rats sham-operated group (NS); (ii) nondiabetic rats I/R group (NI/R); (iii) diabetic rats sham-operated group (DS); (iv) diabetic rats I/R group (DI/R); (v) diabetic rats I/R+melatonin group; and (vi) diabetic rats I/R+melatonin+EX527 group. Melatonin was intraperitoneally injected daily after 3 days of STZ treatment for 4 weeks before renal I/R injury model (10 mg/kg, dissolved in 1% ethanol) [40]. EX527 was intraperitoneally injected daily for 3 days before renal I/R injury and once injected at 20 min before reperfusion (5 mg/kg, 1% DMSO diluted in sterile saline) [41].

### Renal function and histology

Blood urea nitrogen (BUN) and serum creatinine (Scr) were measured by using commercial kits (Jiancheng Biotech, Nanjing, China) to detect renal function. Kidney tissues were cut into sections and fixed with 4% formaldehyde for 24 h, dehydrated and embedded in paraffin following routine protocols. After embedding in paraffin, 4-μm-thick sections were stained with Hematoxylin at room temperature for 3 min and Eosin for 60 s using light microscopy.

Histopathological changes were evaluated by the degree of tubular injury graded from 0 to 4, according to tubular epithelial cell swelling, interstitial expansion, intertubular hemorrhaging, brush border loss, vacuolar degeneration, necrotic tubules, cast formation, and desquamation. Each sample was quantitated by five randomly selected fields with the following criteria: 0, no damage; 1, <25%; 2, 25–50%; 3, 50–75%; 4, >75%. Histological sections were evaluated in a blinding manner by two examiners [42].

### Apoptosis assay

Terminal-deoxynucleoitidyl Transferase Mediated Nick End Labeling (TUNEL) was used to detect kidney tissue apoptosis using an *in situ* cell death detection kit (Roche Diagnostics, Mannheim, Germany). Briefly, paraffin sections routinely underwent deparaffinization and rehydration, and then the slides were treated with 20 mg/l of proteinase K at 37°C for 15–25 min. The slides were then washed in PBS, the mass concentration of 3 g/l hydrogen peroxide/methanol was used to block endogenous peroxidase activity for 30 min at room temperature. The slides were then washed in PBS and then added to the TUNEL reaction mixture for 60 min in a humidified atmosphere at 37°C in the dark. The steps including washing in PBS, adding converter-POD, and incubating at 37°C for 30 min were then performed. Then, the slides were washed in PBS, and Diaminobenzidine (DAB) staining was performed. In addition, Hematoxylin was selected for re-staining. Finally, dehydration and transparent treatment were performed. TUNEL-positive cells were stained brown within the nucleus of apoptotic cells. Cell counting was performed by using five randomly selected fields, and the apoptosis index was calculated as the percentage of positive cells to total cells.

### Measurement of oxidative stress

The level of malondialdehyde (MDA) and superoxide dismutase (SOD) from the homogenized kidney tissue was measured by using commercial kits respectively (Jiancheng Biotech, Nanjing, China), according to the manufacturer’s instructions.

### Western blot analysis

Cytoplasmic and nuclear proteins were extracted from the renal tissues using a nuclear extraction kit (Beyotime Institute of Biotechnology, Haimen, China) according to the manufacturer’s instructions. The expressions of SIRT1, Nrf2, and HO-1 were examined by Western blot. GAPDH was used as the internal loading control of cytoplasmic protein. Lamin B was used as the internal loading control of nuclear protein. Protein content was determined by BCA protein assay kit (Beyotime Institute of Biotechnology, China). Protein samples were separated by electrophoresis on SDS/PAGE and transferred to PVDF membranes (Millipore, Billerica, MA, U.S.A.). Each membrane was blocked with 5% nonfat milk and incubated overnight at 4°C with the appropriate primary antibodies (1:1000 dilution, anti-SIRT1 and anti-HO-1 antibody, 1:500 dilution, anti-Nrf2 antibody), respectively followed by incubation with suitable secondary antibodies for 1 h at room temperature. Immune complexes were detected by using an Odyssey fluorescence-imaging scanner and band densities were quantitated using Odyssey software v3.0.29 imaging analysis system (both from LI-COR Biosciences, Lincoln, NE, U.S.A.).

### Statistical analysis

All data were expressed as the mean ± S.E.M. and analyzed using GraphPad Prism software version 6.0 (GraphPad Software, Inc., La Jolla, CA, U.S.A.). The statistical significance of differences amongst control and diabetic rats were evaluated by one-way ANOVA or two-way ANOVA followed by a Bonferroni’s post hoc test. *P*-values <0.05 were considered to be statistically significant.

## Results

### Characteristics of control and diabetic rats before I/R modeling

At the end of the present study, the diabetic rats showed obvious characteristic systems of diabetes including hyperglycemia, polydipsia, polyphagia, and weight loss. Compared with the age-matched nondiabetic rats, the blood glucose of diabetic rats was significantly increased, and their body weight was significantly reduced (Table 1). Melatonin treatment had no significant effects on blood glucose and body weight in diabetic rats (Table 1).

**Table 1.** Fasting blood glucose levels and body weight of nondiabetic and diabetic rats after 4 weeks

	NS	NI/R	DS	DI/R	DI/R+melatonin	DI/R+melatonin+ EX527
Fasting blood glucose (mM)	5.88 ± 0.88	7.11 ± 1.61	25.51 ± 2.73*	27.19 ± 2.38*	24.45 ± 2.27*	26.21 ± 1.90*
Body weight (g)	345.69 ± 13.01	354.5 ± 9.98	206.06 ± 9.28*	213.76 ± 12.56*	221.12 ± 10.63*	209.32 ± 13.29*

The data are expressed as means ± S.E.M. (*n*=6–8 per group). NS and DS: nondiabetic and diabetic rats were subjected to sham operation. NI/R and DI/R: nondiabetic and diabetic rats were subjected to 30 min bilateral renal pedicle ligation and followed by 48 h reperfusion. DIR+melatonin group: diabetic rats subjected to I/R surgery were treated with melatonin (10 mg/kg, ip daily) for 4 weeks after 3 days of STZ treatment. DIR+melatonin+EX527 group: diabetic rats subjected to I/R operation were treated with melatonin (10 mg/kg, ip daily) for 4 weeks after 3 days of STZ treatment, and treated with EX527 for 3 days before renal I/R injury model and once injected at 20 min before reperfusion (5 mg/kg, ip daily). *P<0.05 compared with NS group and NI/R group.

### Diabetic rats exhibit aggravated ischemia AKI-induced kidney injury on histopathology and apoptosis

We compared the susceptibility of diabetic and nondiabetic rats with I/R. The tubular injury score was used to evaluate the severity of kidney injury. Pathological changes were observed in renal tubules, including tubular epithelial cell swelling, brush border loss, interstitial expansion, intertubular hemorrhaging, vacuolar degeneration, necrotic tubules, cast formation, and desquamation in the NI/R group and diabetic groups (Figure 1A,C). A significant aggravating tissue damage was also observed in DI/R group (Figure 1A,C). When compared with the sham group, the NI/R group and diabetic groups exhibited a significant increase in histopathological scoring individually (*P*<0.05; Figure 1A,C). Moreover, a TUNEL assay was performed to identify the apoptotic cells in renal tissues. The TUNEL-positive cells were diminished in both NS and DS groups (Figure 1B). After I/R for 48 h, the apoptosis index of DI/R group was significantly higher than NI/R group (*P*<0.05; Figure 1D).

**Figure 1:** A diabetic model of adult male SD rats was induced using STZ All rats were subjected to sham surgery or bilateral renal I/R injury. (**A**) Renal Hematoxylin and Eosin staining. Magnification: 200×. The lower panels are the magnified images of the boxed areas in the upper panels. (**B**) TUNEL staining. Magnification: 400×. (**C**) Histopathological scoring. (**D**) TUNEL assay apoptosis%. Data are presented as the mean ± S.E.M. (*n*=6 per group). ^★^*P*<0.05 compared with NS group; ^▲^*P*<0.05 compared with NI/R group; ^#^*P*<0.05 compared with DS group. Abbreviations: Ctrl, control; DM, diabetes mellitus; HE, Hematoxylin and Eosin.

### Diabetic rats exhibit aggravated kidney dysfunction and increased oxidative stress in the kidney after ischemia AKI

Diabetic I/R injury aggravated renal damage and oxidative stress [43]. Compared with the NS and DS groups, the levels of the BUN and SCr were significantly increased 48 h post I/R in both the NI/R and DI/R groups (*P*<0.05; Figure 2A,B). The damage evoked by AKI was further increased in the DI/R group, demonstrated by higher levels of the BUN and Scr than NI/R group (*P*<0.05; Figure 2A,B). In addition, as an indicator of antioxidant, SOD levels were significantly decreased in the NI/R and DI/R groups as compared with the NS and DS groups, respectively (*P*<0.05; Figure 2C). Meanwhile, the SOD level in DI/R group was lower than the NI/R group (*P*<0.05; Figure 2C). In contrast, the level of MDA, used as a measure of the level of oxidative stress, was significantly increased in the NI/R and DI/R groups, compared with those in the NS and DS groups, respectively (*P*<0.05; Figure 2D). When compared with NI/R group, the MDA level was significantly higher in DI/R group (*P*<0.05; Figure 2D).

**Figure 2:** Serum BUN, creatinine, and renal tissues SOD and MDA levels in the different treatment groups (**A**) BUN. (**B**) Scr. (**C**) Kidney SOD contents. (**D**) MDA activity. Data are presented as the mean ± S.E.M. (*n*=6 per group). ^★^*P*<0.05 compared with NS group; ^▲^*P*<0.05 compared with NI/R group; ^#^*P*<0.05 compared with DS group. Abbreviations: Ctrl, control; DM, diabetes mellitus.

### Protein expression of SIRT1, Nrf2, and HO-1 in renal tissues

The previous research showed that the expression of SIRT1 is significantly reduced in DKI [44]. Similarly, the protein expression of SIRT1 was significantly diminished in DS group compared with NS group (*P*<0.05; Figure 3A,C). Renal SIRT1 expression was increased in NI/R group compared with NS group (*P*<0.05; Figure 3A,C). Renal SIRT1 expression was decreased in DI/R group compared with DS group (*P*<0.05; Figure 3A,C). Furthermore, the expression of SIRT1 was decreased in DI/R group compared with NI/R group (*P*<0.05; Figure 3A,C). The Nrf2/HO-1 pathway plays an important role in antioxidant reaction [45,46]. We detected the expression of Nrf2 and HO-1 in all groups. The results revealed that Nrf2 and HO-1 expression was diminished in DS and DI/R groups, compared with NS group, respectively. A significant increase in Nrf2 and HO-1 were observed in the NI/R group, when compared with NS group. Renal expression of Nrf2 and HO-1 were both decreased in DI/R group compared with NI/R group and DS group respectively (*P*<0.05; Figure 3A,B,D).

**Figure 3:** Expression of SIRT1, Nrf2, and HO-1 in renal tissues by Western blot analysis (**A**) Western blotting showed protein levels of SIRT1, Nrf2, and HO-1. (**B**–**D**) Quantitation of Western blot data from (A). Data are presented as the mean ± S.E.M. (*n*=6 per group). ^★^*P*<0.05 compared with NS group; ^▲^*P*<0.05 compared with NI/R group; ^#^*P*<0.05 compared with DS group. Abbreviations: Ctrl, control; DM, diabetes mellitus.

### Effects of melatonin on histopathology and apoptosis

Ischemia induces NO synthase in tubule cells. Subsequently, ROS cause renal tubule cell injury via oxidation of proteins, peroxidation of lipids, damage to DNA, and induction of apoptosis [47]. After I/R occurred, C3 deposited in renal and injured tubular epithelial cells, subsequently led to apoptosis due to the lack of the decay accelerating factor (DAF) and membrane cofactor protein (MCP) which inhibit complement activation of C3/4 level that is located in glomerular, rather tubular [48,49]. Melatonin exhibited anti-apoptosis in STZ-induced diabetic renal injury [50], as well as in I/R injury in the model of experimental kidney transplantation [16]. However, whether melatonin remains anti-apoptotic and how it affects the histopathology in the kidney is still unknown. Interestingly, the pathological changes in renal tubules, histopathological scoring, and apoptotic index were significantly increased in DI/R group and DI/R+melatonin+EX527 group, as compared with DS group (*P*<0.05; Figure 4A–D), while melatonin pre-treatment markedly ameliorated the histology score and apoptosis in DI/R+melatonin group, compared with the DI/R group and DI/R+melatonin+EX527 group (*P*<0.05; Figure 4C,D). Pre-treatment with EX527 in DI/R+melatonin+EX527 group abolished the positive effects elicited by melatonin (*P*<0.05; Figure 4C,D). There was no statistically significant difference in histopathological scoring and apoptotic index between DI/R group and DI/R+melatonin+EX527 group (*P*>0.05; Figure 4C,D).

**Figure 4:** Melatonin pre-treatment markedly ameliorated the histology score and apoptosis after bilateral renal I/R injury in diabetic rats (**A**) Renal HE staining. Magnification: 200×. The lower panels are the magnified images of the boxed areas in the upper panels. (**B**) TUNEL staining. Magnification: 400×. (**C**) Histopathological scoring. (**D**) TUNEL assay apoptosis%. Data are presented as the mean ± S.E.M. (*n*=6 per group). ^★^*P*<0.05 compared with DS group; ^▲^*P*<0.05 compared with DI/R+melatonin group. Abbreviation: HE, Hematoxylin and Eosin.

### Melatonin attenuates kidney dysfunction and oxidative stress in the kidney after ischemia AKI

Both diabetes or I/R injury aggravated kidney dysfunction and oxidative stress that could be reversed by melatonin treatment [50,51]. In our study, melatonin significantly decreased the BUN and Scr in DI/R+melatonin group compared with DI/R group and DI/R+melatonin+EX527 group (*P*<0.05; Figure 5A,B). EX527 pre-treatment abolished the positive effects on BUN and Scr elicited by melatonin (*P*<0.05; Figure 5A,B). We next examined the effect of melatonin on SOD and MDA levels. Compared with DI/R group and DI/R+melatonin+EX527 group, SOD activity was significantly increased in DI/R+melatonin, while the effect was abolished by EX527 in DI/R+melatonin+EX527 group (*P*<0.05; Figure 5C). The MDA production in the melatonin-treated group was significantly decreased, compared with DI/R group and DI/R+melatonin+EX527 group (*P*<0.05; Figure 5D). Meanwhile, the melatonin-induced reduction in MDA level was abolished by EX527 in DI/R+melatonin+EX527 group (*P*<0.05; Figure 5D).

**Figure 5:** Melatonin pre-treatment attenuates kidney dysfunction and oxidative stress after I/R injury in diabetic rats (**A**) BUN. (**B**) Scr. (**C**) Kidney SOD contents. (**D**) MDA activity. Data are presented as the mean ± S.E.M. (*n*=6 per group). ^★^*P*<0.05 compared with DS group; ^▲^*P*<0.05 compared with DI/R+melatonin group.

### Effects of melatonin on protein expression of SIRT1, Nrf2, and HO-1 in renal tissues

The activation of SIRT1 was observed in AKI [52]. We detected SIRT1 in all groups and found that protein expression of SIRT1 was significantly reduced in the DI/R group compared with the DS group (*P*<0.05; Figure 6A,C). Melatonin administration significantly increased SIRT1 expression in DI/R+melatonin group compared with the DI/R group, whereas EX527 eliminated this effect in the DI/R+melatonin+EX527 group (*P*<0.05; Figure 6A,C). There was no significant difference in the expression of SIRT1 between the DI/R group and the DI/R+melatonin+EX527 group (*P*>0.05; Figure 6A,C). The protective effects of melatonin in I/R injury are relative to antioxidative stress rather than the pro-inflammatory cytokines [21,22]. Meanwhile melatonin attenuates cisplatin-induced nephrotoxicity by increasing the expression of Nrf2 and HO-1 [53]. We then examined the protein expression of Nrf2 and HO-1 after AKI, and the expression of Nrf2 and HO-1 was decreased in the DI/R group compared with the DS group (*P*<0.05; Figure 6A,B,D). The levels of Nrf2 and HO-1 in DI/R+melatonin group were significantly increased compared with the DI/R group, respectively (*P*<0.05; Figure 6A,B,D). However, the use of EX527 in the DI/R+melatonin+EX527 group abolished the increased expression of Nrf2 and HO-1 compared with DI/R+melatonin group (*P*<0.05; Figure 6A,B,D). There was no significant difference in the expression of Nrf2 and HO-1 between the DI/R group and the DI/R+melatonin+EX527 group (*P*>0.05; Figure 6A,B,D).

**Figure 6:** Melatonin pre-treatment up-regulates SIRT1, Nrf2, and HO-1 expression after kidney I/R injury in diabetic rats (**A**) Western blotting showed protein levels of SIRT1, Nrf2, and HO-1. (**B**–**D**) Quantitation of Western blot data from (A). Data are presented as the mean ± S.E.M. (*n*=6 per group). ^★^*P*<0.05 compared with DS group; ^▲^*P*<0.05 compared with DI/R+melatonin group.

## Discussion

Diabetes is a potential risk factor for increasing AKI and mortality/morbidity of AKI [54]. One of the major risk factors for AKI is the I/R injury. Ischemia-induced AKI after kidney transplant surgery, secondary to I/R injury, is a major factor affecting both short-term and long-term grafts and patient survival [55]. Previous studies have shown that increased diabetic kidney I/R susceptibility correlates with oxidative stress and nitrification stress [56]. A recent study showed that diabetic rats undergoing I/R can increase apoptosis, BUN, and Scr levels, and the decreased tolerance to I/R in diabetic rats may be associated with increased pro-inflammatory cytokines [7]. Consistent with previous studies, we found that diabetes aggravated renal I/R injury through the pathological changes in renal tubules. Meanwhile, diabetes dramatically increased I/R-induced cell apoptosis [6]. As known previously, I/R induced kidney dysfunction and on this basis, diabetes remarkably exacerbated the damage in kidney function reflected in the higher levels of BUN and Scr. In addition, the change of SOD, an indicator of antioxidant, was lower in both NI/R and DI/R groups, especially in DI/R group, and MDA, as an indicator of oxidative stress that was higher in both NI/R and DI/R groups, especially in DI/R group, we speculated that all the above effects are caused by enhanced oxidative stress and diabetes further aggravated it on the basis of I/R injury. Our findings are consistent with previous studies [6,7].

Previous studies have verified that SIRT1, an NAD^+^-dependent histone deacetylase, plays a positive role in type 2 diabetes mellitus (T2DM) with the function of anti-oxygenation and anti-inflammation [57]. Meanwhile the activation of SIRT1 promoted Nrf2 nuclear translocation and anti-oxygenation in the situation of diabetic MI/R injury [58]. And activating Nrf2/HO-1 pathway alleviates renal I/R injury in diabetic rats [59]. Our results showed that, in the condition of diabetic AKI, the expression of SIRT1 was decreased, and Nrf2/HO-1 pathway was inhibited. However, the Nrf2/HO-1 pathway was activated by melatonin through activating SIRT1.

Melatonin is anti-inflammatory, antioxidative, and reduces endoplasmic reticulum stress in the AKI [60–62]. The previous study has reported that melatonin reduces kidney injury by reducing lipid oxidation and NO production in STZ-induced diabetic rats [15]. In our research, we found melatonin ameliorated the histopathological scoring, alleviated apoptotic index, reduced the levels of BUN and Scr, decreased MDA, and increased SOD in DI/R+melatonin group, while this effect was eliminated by EX527, a SIRT1 inhibitor. However, the mechanism of melatonin treatment to reduce AKI in diabetes has not been reported yet. In the present study, we provided evidence that diabetic rats exhibited enhanced kidney histological damage, increased kidney apoptosis, aggravated kidney dysfunction, and elevated oxidative stress after AKI injury. However, melatonin administration attenuated these unfavorable results. Previous studies have shown that the melatonin protects the function of kidney and brain by effecting SIRT1, as well as in diabetic heart [33,63–65]. Our study showed that treatment with melatonin, restores the expression of SIRT1 that could further enhance expression of Nrf2 and HO-1, compared with the DI/R group. While EX527 reversed the changes of Nrf2 and HO-1 induced by SIRT1, suggesting melatonin could protect kidney against I/R injury in diabetes by up-regulating the expression of the SIRT1 protein, which then consequently activates Nrf2 and induce HO-1 expression.

A study has reported that activating SIRT1 could stabilize the transcription factor Nrf2 by its deacetylation [66]. Up-regulating the SIRT1-Nrf2 signaling pathway can reduce oxidative stress and inflammation [67]. Another study in experimental traumatic brain injury reported that melatonin can affect the expression of NRF2 and HO-1, but its mechanism needs further investigation [68]. However, a recent study confirmed that melatonin attenuates lipopolysaccharide-induced oxidative stress in rat brain by activating the SIRT1/Nrf2 signaling pathway [69]. In our study, we found that diabetes aggravate kidney apoptosis, kidney dysfunction, and oxidative stress after AKI injury. Melatonin reduced the kidney damage caused by diabetes and I/R injury, however, EX527 abolished the protective effect of melatonin. We further investigated how melatonin and EX527 influence the diabetic kidney that underwent I/R injury and found that melatonin could change the amount of Nrf2 and HO-1 through influencing the expression of SIRT1, at the same time EX527 blocking the activation of Nrf2/HO-1 pathway by inhibiting the SIRT1 expression. According to our findings, we suggest that melatonin protects diabetes kidney by activating SIRT1/Nrf2/HO-1 pathway.

## Conclusion

Taken together, our findings indicate that hyperglycemia-induced oxidative stress is involved in impaired SIRT1/Nrf2/HO-1 signaling and ischemia AKI in diabetes. Inhibition of oxidative stress with melatonin attenuates ischemia AKI in diabetes by improving the SIRT1/Nrf2/HO-1 signaling. Melatonin attenuates apoptosis and oxidative stress in diabetes ischemia AKI through activation of the SIRT1/Nrf2/HO-1 pathway. Moreover, its beneficial effects on heart and brain in diabetes may make melatonin a potential therapeutic drug especially under the condition of I/R. In addition, SIRT1/Nrf2/HO-1 pathway could be a new target in decreasing the oxidative stress in diabetic I/R injury.

## Abbreviations

AKI: acute kidney injury
Akt: Protein Kinase B
ARE: antioxidant response elements
BUN: blood urea nitrogen
DI/R: diabetic rats ischemia/reperfusion
DKI: diabetic kidney injury
DN: diabetic nephropathy
DS: diabetic rats sham-operated
GAPDH: glyceraldehyde-3-phosphate dehydrogenase
GSK-3β: Glycogen synthase kinase-3 beta
HO-1: heme oxygenase-1
I/R: ischemia/reperfusion
iNOS: nitric oxide synthase
MDA: malondialdehyde
NF-kBp65: nuclear factor-kappa B p65
NI/R: nondiabetic rats ischemia/reperfusion
NQO1: NADPH Quinone oxidoreductase 1
Nrf2: nuclear factor erythroid 2-related factor 2
NS: nondiabetic rats sham-operated
POD: peroxidase
ROS: reactive oxygen species
Scr: serum creatinine
SIRT1: silent information regulator 2 associated protein 1
SOD: superoxide dismutase
STZ: streptozotocin
TUNEL: terminal-deoxynucleoitidyl transferase mediated nick end labeling
VDAC: Voltage-dependent anion channel

## References

[1] BaoY.W., YuanY., ChenJ.H. and LinW.Q. (2018) Kidney disease models: tools to identify mechanisms and potential therapeutic targets. Zool. Res. 39, 72–86 2951508910.24272/j.issn.2095-8137.2017.055PMC5885387

[2] YuS.M. and BonventreJ.V. (2018) Acute kidney injury and progression of diabetic kidney disease. Adv. Chronic Kidney Dis. 25, 166–180 10.1053/j.ackd.2017.12.005 29580581PMC5898826

[3] MacIsaacR.J., JerumsG. and EkinciE.I. (2018) Glycemic control as primary prevention for diabetic kidney disease. Adv. Chronic Kidney Dis. 25, 141–148 10.1053/j.ackd.2017.11.003 29580578

[4] GiuntiS., BaritD. and CooperM.E. (2006) Diabetic nephropathy: from mechanisms to rational therapies. Minerva Med. 97, 241–262 16855519

[5] AghadavodE., KhodadadiS., BaradaranA., NasriP., BahmaniM. and Rafieian-KopaeiM. (2016) Role of oxidative stress and inflammatory factors in diabetic kidney disease. Iran J. Kidney Dis. 10, 337–343 27903991

[6] XiaoY.D., HuangY.Y., WangH.X., WuY., LengY., LiuM. (2016) Thioredoxin-interacting protein mediates NLRP3 inflammasome activation involved in the susceptibility to ischemic acute kidney injury in diabetes. Oxid. Med. Cell Longev. 2016, 2386068 10.1155/2016/2386068 27867451PMC5102753

[7] ZhangY., HuF., WenJ., WeiX., ZengY., SunY. (2017) Effects of sevoflurane on NF-small ka, CyrillicB and TNF-alpha expression in renal ischemia-reperfusion diabetic rats. Inflamm. Res. 66, 901–910 10.1007/s00011-017-1071-1 28685196

[8] TanD.X., HardelandR., BackK., ManchesterL.C., Alatorre-JimenezM.A. and ReiterR.J. (2016) On the significance of an alternate pathway of melatonin synthesis via 5-methoxytryptamine: comparisons across species. J. Pineal Res. 61, 27–40 10.1111/jpi.12336 27112772

[9] TordjmanS., ChokronS., DelormeR., CharrierA., BellissantE., JaafariN. (2017) Melatonin: pharmacology, functions and therapeutic benefits. Curr. Neuropharmacol. 15, 434–443 10.2174/1570159X14666161228122115 28503116PMC5405617

[10] ReiterR.J. and TanD.X. (2003) Melatonin: a novel protective agent against oxidative injury of the ischemic/reperfused heart. Cardiovasc. Res. 58, 10–19 10.1016/S0008-6363(02)00827-1 12667942

[11] SuzenS., BozkayaP., CobanT. and NebioguD. (2006) Investigation of the in vitro antioxidant behaviour of some 2-phenylindole derivatives: discussion on possible antioxidant mechanisms and comparison with melatonin. J. Enzyme Inhib. Med. Chem. 21, 405–411 10.1080/14756360500381210 17059173

[12] HardelandR. (2005) Antioxidative protection by melatonin: multiplicity of mechanisms from radical detoxification to radical avoidance. Endocrine 27, 119–130 10.1385/ENDO:27:2:119 16217125

[13] Tomas-ZapicoC. and Coto-MontesA. (2005) A proposed mechanism to explain the stimulatory effect of melatonin on antioxidative enzymes. J. Pineal Res. 39, 99–104 10.1111/j.1600-079X.2005.00248.x 16098085

[14] EspinoJ., RodriguezA.B. and ParienteJ.A. (2018) Melatonin and oxidative stress in the diabetic state: clinical implications and potential therapeutic applications. Curr. Med. Chem., 25, 1–11 10.2174/0929867325666180410094149 29637854

[15] KurcerZ., ParlakpinarH., VardiN., TasdemirS., IrazM., FadilliogluE. (2007) Protective effects of chronic melatonin treatment against renal ischemia/reperfusion injury in streptozotocin-induced diabetic rats. Exp. Clin. Endocrinol. Diabetes 115, 365–371 10.1055/s-2007-971056 17701881

[16] LiZ., NickkholghA., YiX., BrunsH., GrossM.L., HoffmannK. (2009) Melatonin protects kidney grafts from ischemia/reperfusion injury through inhibition of NF-kB and apoptosis after experimental kidney transplantation. J. Pineal Res. 46, 365–372 10.1111/j.1600-079X.2009.00672.x 19552759

[17] HadjA.T.K., MahfoudhB.A., ZaoualiM.A., KammounR., BejaouiM., GhoulM.S. (2015) Melatonin modulates endoplasmic reticulum stress and Akt/GSK3-beta signaling pathway in a rat model of renal warm ischemia reperfusion. Anal. Cell Pathol. (Amst.) 2015, 635172 2622974310.1155/2015/635172PMC4502281

[18] LongT., YangY., PengL. and LiZ. (2018) Neuroprotective effects of melatonin on experimental allergic encephalomyelitis mice via anti-oxidative stress activity. J. Mol. Neurosci. 64, 233–241 10.1007/s12031-017-1022-x 29450696

[19] Carrillo-VicoA., LardoneP.J., Alvarez-SanchezN., Rodriguez-RodriguezA. and GuerreroJ.M. (2013) Melatonin: buffering the immune system. Int. J. Mol. Sci. 14, 8638–8683 10.3390/ijms14048638 23609496PMC3645767

[20] ZubidatA.E., NelsonR.J. and HaimA. (2010) Photoentrainment in blind and sighted rodent species: responses to photophase light with different wavelengths. J. Exp. Biol. 213, 4213–4222 10.1242/jeb.048629 21113002

[21] KurcerZ., OguzE., OzbilgeH., BabaF., AksoyN. and CelikN. (2008) Effect of melatonin on testicular ischemia/reperfusion injury in rats: is this effect related to the proinflammatory cytokines? Fertil. Steril. 89, 1468–1473 10.1016/j.fertnstert.2007.04.065 17681337

[22] KurcerZ., OguzE., OzbilgeH., BabaF., AksoyN., CelikH. (2007) Melatonin protects from ischemia/reperfusion-induced renal injury in rats: this effect is not mediated by proinflammatory cytokines. J. Pineal Res. 43, 172–178 10.1111/j.1600-079X.2007.00459.x 17645695

[23] Martinez-RedondoP. and VaqueroA. (2013) The diversity of histone versus nonhistone sirtuin substrates. Genes Cancer 4, 148–163 10.1177/1947601913483767 24020006PMC3764476

[24] BonkowskiM.S. and SinclairD.A. (2016) Slowing ageing by design: the rise of NAD(+) and sirtuin-activating compounds. Nat. Rev. Mol. Cell Biol. 17, 679–690 10.1038/nrm.2016.93 27552971PMC5107309

[25] RahmanS. and IslamR. (2011) Mammalian Sirt1: insights on its biological functions. Cell Commun. Signal 9, 11 10.1186/1478-811X-9-11 21549004PMC3103488

[26] VaziriH., DessainS.K., NgE.E., ImaiS.I., FryeR.A., PanditaT.K. (2001) hSIR2(SIRT1) functions as an NAD-dependent p53 deacetylase. Cell 107, 149–159 10.1016/S0092-8674(01)00527-X 11672523

[27] DaitokuH., HattaM., MatsuzakiH., ArataniS., OhshimaT., MiyagishiM. (2004) Silent information regulator 2 potentiates Foxo1-mediated transcription through its deacetylase activity. Proc. Natl. Acad. Sci. U.S.A. 101, 10042–10047 10.1073/pnas.040059310115220471PMC454161

[28] YeungF., HobergJ.E., RamseyC.S., KellerM.D., JonesD.R., FryeR.A. (2004) Modulation of NF-kappaB-dependent transcription and cell survival by the SIRT1 deacetylase. EMBO J. 23, 2369–2380 10.1038/sj.emboj.7600244 15152190PMC423286

[29] HaigisM.C. and SinclairD.A. (2010) Mammalian sirtuins: biological insights and disease relevance. Annu. Rev. Pathol. 5, 253–295 10.1146/annurev.pathol.4.110807.092250 20078221PMC2866163

[30] KumeS., KitadaM., KanasakiK., MaegawaH. and KoyaD. (2013) Anti-aging molecule, Sirt1: a novel therapeutic target for diabetic nephropathy. Arch. Pharm. Res. 36, 230–236 10.1007/s12272-013-0019-4 23361587

[31] KitadaM., KumeS., Takeda-WatanabeA., KanasakiK. and KoyaD. (2013) Sirtuins and renal diseases: relationship with aging and diabetic nephropathy. Clin. Sci. (Lond.) 124, 153–164 10.1042/CS20120190 23075334PMC3466784

[32] GuanY. and HaoC.M. (2016) SIRT1 and kidney function. Kidney Dis. 1, 258–265 10.1159/000440967 27536685PMC4934818

[33] BaiX.Z., HeT., GaoJ.X., LiuY., LiuJ.Q., HanS.C. (2016) Melatonin prevents acute kidney injury in severely burned rats via the activation of SIRT1. Sci. Rep. 6, 32199 10.1038/srep32199 27599451PMC5013284

[34] JiangT., TianF., ZhengH., WhitmanS.A., LinY., ZhangZ. (2014) Nrf2 suppresses lupus nephritis through inhibition of oxidative injury and the NF-kappaB-mediated inflammatory response. Kidney Int. 85, 333–343 10.1038/ki.2013.343 24025640PMC3992978

[35] SheltonL.M., ParkB.K. and CoppleI.M. (2013) Role of Nrf2 in protection against acute kidney injury. Kidney Int. 84, 1090–1095 10.1038/ki.2013.248 23783243

[36] HuangK., GaoX. and WeiW. (2017) The crosstalk between Sirt1 and Keap1/Nrf2/ARE anti-oxidative pathway forms a positive feedback loop to inhibit FN and TGF-beta1 expressions in rat glomerular mesangial cells. Exp. Cell Res. 361, 63–72 10.1016/j.yexcr.2017.09.042 28986066

[37] HuangK., ChenC., HaoJ., HuangJ., WangS., LiuP. (2015) Polydatin promotes Nrf2-ARE anti-oxidative pathway through activating Sirt1 to resist AGEs-induced upregulation of fibronetin and transforming growth factor-beta1 in rat glomerular messangial cells. Mol. Cell Endocrinol. 399, 178–189 2519279710.1016/j.mce.2014.08.014

[38] HuangK., LiR. and WeiW. (2018) Sirt1 activation prevents anti-Thy 1.1 mesangial proliferative glomerulonephritis in the rat through the Nrf2/ARE pathway. Eur. J. Pharmacol. 832, 138–144 2978285610.1016/j.ejphar.2018.05.017

[39] XueR., LeiS., XiaZ.Y., WuY., MengQ., ZhanL. (2016) Selective inhibition of PTEN preserves ischaemic post-conditioning cardioprotection in STZ-induced Type 1 diabetic rats: role of the PI3K/Akt and JAK2/STAT3 pathways. Clin. Sci. (Lond.) 130, 377–392 2666644410.1042/CS20150496

[40] VuralH., SabuncuT., ArslanS.O. and AksoyN. (2001) Melatonin inhibits lipid peroxidation and stimulates the antioxidant status of diabetic rats. J. Pineal Res. 31, 193–198 1158975210.1034/j.1600-079x.2001.310301.x

[41] YuL., LiS., TangX., LiZ., ZhangJ., XueX. (2017) Diallyl trisulfide ameliorates myocardial ischemia-reperfusion injury by reducing oxidative stress and endoplasmic reticulum stress-mediated apoptosis in type 1 diabetic rats: role of SIRT1 activation. Apoptosis 22, 942–954 2845582410.1007/s10495-017-1378-y

[42] YangK., LiW.F., YuJ.F., YiC. and HuangW.F. (2017) Diosmetin protects against ischemia/reperfusion-induced acute kidney injury in mice. J. Surg. Res. 214, 69–782862406210.1016/j.jss.2017.02.067

[43] HuB., TongF., XuL., ShenZ., YanL., XuG. (2018) Role of calcium sensing receptor in streptozotocin-induced diabetic rats exposed to renal ischemia reperfusion injury. Kidney Blood Press. Res. 43, 276–2862949030610.1159/000487685

[44] ChuangP.Y., DaiY., LiuR., HeH., KretzlerM., JimB. (2011) Alteration of forkhead box O (foxo4) acetylation mediates apoptosis of podocytes in diabetes mellitus. PLoS ONE 6, e23566 2185816910.1371/journal.pone.0023566PMC3157434

[45] ShokeirA.A., BarakatN., HusseinA.M., AwadallaA., HarrazA.M., KhaterS. (2015) Activation of Nrf2 by ischemic preconditioning and sulforaphane in renal ischemia/reperfusion injury: a comparative experimental study. Physiol. Res. 64, 313–323 2553631910.33549/physiolres.932834

[46] ZhangY., RongS., FengY., ZhaoL., HongJ., WangR. (2017) Simvastatin attenuates renal ischemia/reperfusion injury from oxidative stress via targeting Nrf2/HO-1 pathway. Exp. Ther. Med. 14, 4460–4466 2906712010.3892/etm.2017.5023PMC5647698

[47] DevarajanP. (2006) Update on mechanisms of ischemic acute kidney injury. J. Am. Soc. Nephrol. 17, 1503–1520 10.1681/ASN.2006010017 16707563

[48] De VriesB., MatthijsenR.A., WolfsT.G., Van BijnenA.A., HeeringaP. and BuurmanW.A. (2003) Inhibition of complement factor C5 protects against renal ischemia-reperfusion injury: inhibition of late apoptosis and inflammation. Transplantation 75, 375–382 10.1097/01.TP.0000044455.05584.2A 12589162

[49] IchidaS., YuzawaY., OkadaH., YoshiokaK. and MatsuoS. (1994) Localization of the complement regulatory proteins in the normal human kidney. Kidney Int. 46, 89–96 10.1038/ki.1994.247 7523758

[50] MotawiT.K., AhmedS.A., A HamedM., El-MaraghyS.A. and M AzizW. (2017) Melatonin and/or rowatinex attenuate streptozotocin-induced diabetic renal injury in rats. J. Biomed. Res., [Epub ahead of print] 10.7555/JBR.31.20160028 29089475PMC6477174

[51] KunduzovaO.R., EscourrouG., SeguelasM.H., DelagrangeP., De La FargeF., CambonC. (2003) Prevention of apoptotic and necrotic cell death, caspase-3 activation, and renal dysfunction by melatonin after ischemia/reperfusion. FASEB J. 17, 872–874 10.1096/fj.02-0504fje 12670883

[52] BaiX.Z., HeT., GaoJ.X., LiuY., LiuJ.Q., HanS.C. (2016) Melatonin prevents acute kidney injury in severely burned rats via the activation of SIRT1. Sci. Rep. 6, 32199 10.1038/srep32199 27599451PMC5013284

[53] KilicU., KilicE., TuzcuZ., TuzcuM., OzercanI.H., YilmazO. (2013) Melatonin suppresses cisplatin-induced nephrotoxicity via activation of Nrf-2/HO-1 pathway. Nutr. Metab. (Lond.) 10, 7 10.1186/1743-7075-10-723311701PMC3561216

[54] PatschanD. and MullerG.A. (2016) Acute kidney injury in diabetes mellitus. Int. J. Nephrol. 2016, 6232909 10.1155/2016/6232909 27974972PMC5126418

[55] PanahF., GhorbanihaghjoA., ArganiH., AsadiZ.M. and NazariS.A.S. (2018) Ischemic acute kidney injury and klotho in renal transplantation. Clin. Biochem. 55, 3–8 10.1016/j.clinbiochem.2018.03.022 29608890

[56] Abu-SalehN., AwadH., KhamaisiM., ArmalyZ., KarramT., HeymanS.N. (2014) Nephroprotective effects of TVP1022, a non-MAO inhibitor S-isomer of rasagiline, in an experimental model of diabetic renal ischemic injury. Am. J. Physiol. Renal Physiol. 306, F24–F33 10.1152/ajprenal.00379.2013 24197064

[57] KitadaM. and KoyaD. (2013) SIRT1 in type 2 diabetes: mechanisms and therapeutic potential. Diabetes Metab. J. 37, 315–325 10.4093/dmj.2013.37.5.315 24199159PMC3816131

[58] ZhangB., ZhaiM., LiB., LiuZ., LiK., JiangL. (2018) Honokiol ameliorates myocardial ischemia/reperfusion injury in type 1 diabetic rats by reducing oxidative stress and apoptosis through activating the SIRT1-Nrf2 signaling pathway. Oxid. Med. Cell Longev. 2018, 3159801 2967513210.1155/2018/3159801PMC5838504

[59] ShenX., HuB., XuG., ChenF., MaR., ZhangN. (2017) Activation of Nrf2/HO-1 pathway by glycogen synthase kinase-3beta inhibition attenuates renal ischemia/reperfusion injury in diabetic rats. Kidney Blood Press. Res. 42, 369–378 10.1159/000477947 28624830

[60] de SouzaA.V., GolimM.A., DeffuneE., DominguesM.A., de CarvalhoL.R., ViannaI.G. (2014) Evaluation of renal protection from high doses of melatonin in an experimental model of renal ischemia and reperfusion in hyperglycemic rats. Transplant. Proc. 46, 1591–1593 10.1016/j.transproceed.2014.02.024 24834857

[61] OguzE., YilmazZ., OzbilgeH., BabaF., TaburS., YererM.B. (2015) Effects of melatonin on the serum levels of pro-inflammatory cytokines and tissue injury after renal ischemia reperfusion in rats. Renal Fail. 37, 318–322 10.3109/0886022X.2014.991263 25519208

[62] HadjA.T.K., MahfoudhB.A., ZaoualiM.A., KammounR., BejaouiM., GhoulM.S. (2015) Melatonin modulates endoplasmic reticulum stress and Akt/GSK3-beta signaling pathway in a rat model of renal warm ischemia reperfusion. Anal. Cell Pathol. (Amst.) 2015, 635172 2622974310.1155/2015/635172PMC4502281

[63] ZhaoL., LiuH., YueL., ZhangJ., LiX., WangB. (2017) Melatonin attenuates early brain injury via the melatonin receptor/Sirt1/NF-kappaB signaling pathway following subarachnoid hemorrhage in mice. Mol. Neurobiol. 54, 1612–1621 10.1007/s12035-016-9776-7 26867656

[64] ZhaoL., AnR., YangY., YangX., LiuH., YueL. (2015) Melatonin alleviates brain injury in mice subjected to cecal ligation and puncture via attenuating inflammation, apoptosis, and oxidative stress: the role of SIRT1 signaling. J. Pineal Res. 59, 230–239 10.1111/jpi.12254 26094939

[65] YuL., LiangH., DongX., ZhaoG., JinZ., ZhaiM. (2015) Reduced silent information regulator 1 signaling exacerbates myocardial ischemia-reperfusion injury in type 2 diabetic rats and the protective effect of melatonin. J. Pineal Res. 59, 376–390 10.1111/jpi.12269 26327197

[66] DingY.W., ZhaoG.J., LiX.L., HongG.L., LiM.F., QiuQ.M. (2016) SIRT1 exerts protective effects against paraquat-induced injury in mouse type II alveolar epithelial cells by deacetylating NRF2 *in vitro*. Int. J. Mol. Med. 37, 1049–1058 10.3892/ijmm.2016.2503 26935021

[67] DaC.M. and ArrudaS.F. (2017) Tucum-do-Cerrado (Bactris setosa Mart.) may promote anti-aging effect by upregulating SIRT1-Nrf2 pathway and attenuating oxidative stress and inflammation. Nutrients 9, 1243 10.3390/nu9111243PMC570771529135935

[68] DingK., WangH., XuJ., LiT., ZhangL., DingY. (2014) Melatonin stimulates antioxidant enzymes and reduces oxidative stress in experimental traumatic brain injury: the Nrf2-ARE signaling pathway as a potential mechanism. Free Radic. Biol. Med. 73, 1–11 10.1016/j.freeradbiomed.2014.04.031 24810171

[69] ShahS.A., KhanM., JoM.H., JoM.G., AminF.U. and KimM.O. (2017) Melatonin stimulates the SIRT1/Nrf2 signaling pathway counteracting lipopolysaccharide (LPS)-induced oxidative stress to rescue postnatal rat brain. CNS Neurosci. Ther. 23, 33–44 10.1111/cns.12588 27421686PMC6492734

